RETRACTED

# Neuropathological microscopic features of abortions induced by *Bunyavirus */ or *Flavivirus* infections

**DOI:** 10.1186/s13000-014-0223-7

**Published:** 2014-11-26

**Authors:** Javad Javanbakht, Seyed Hossein Mardjanmehr, Abbas Tavasoly, Mohammad Hossein Nazemshirazi

**Affiliations:** 1 Department of Pathology, Faculty of Veterinary Medicine, Tehran University, Tehran, Iran; 2 Department of Molecular Biology, Central Veterinary Laboratory of I.V.O, Tehran, Tehran, Iran

**Keywords:** Lambs, Pathology, Viral infection, Central nervous system malformations, Iran

## Abstract

**Background:**

The present study describes the pathologic changes in the brain and the spinal cord of aborted, stillbirth and deformities of newborn lambs infected with viral agents.

**Methods:**

From February 2012 to March 2013, a total of 650 aborted fetuses from 793 pregnant ewes were studied from 8 flocks at different areas in the Mazandaran province in the north of Iran. And randomly, systematic necropsy was performed to collect tissues, and all gross abnormalities were recorded at necropsy by the pathologist .Nevertheless, we conducted a limited number of necropsies for aborted fetuses.

**Results:**

In the most cases, arthrogryposis was the most common musculoskeletal defects and at necropsy, malformations of the brain included hydranencephaly, porencephaly, hydrocephalus and cerebellar hypoplasia, mainly in the brain stem and gray and white matter of the brain and cerebellum were observed. Histopathologic lesions included chronic multifocal lymphoplasmacytic encephalitis(nonsuppurative) with extensive perivascular cuffing in some cases, formation of glial nodules mainly in the mesencephalon, thalamus, hippocampus, pons and medulla oblongata in the brain of aborted fetuses, and neuronal degeneration, necrosis and central chromatolysis mainly in the cortex and subcortical of the brain and brain stem regions of them. Furthermore, microscopic lesions are mostly linked to a neurodegenerative and necrotic cell death process in the gray matter of ventral horn of the spinal cord. Briefly, histopathologic findings in the brain and spinal cord included hyperemia, hemorrhage, non-suppurative encephalitis, mononuclear perivascular cuffing, multifocal gliosis, cavitation, central chromatolysis, neuronal degeneration and necrosis, perineuronal and perivascular edema in the all regions of the brain and acute neuronal necrosis in the gray matter of ventral horn of the spinal cord were also seen.

**Conclusion:**

Our study suggested that the sheep fetuses are fully susceptible to viral infections and may even develop neurolopathological lesions upon natural infection with mentioned pathogens .Therefore ,according to,specific lesions caused by viral infections, we believe that the histopathological pattern were detected in this study could be associated with either viral infection and or mainly by a *Bunyavirus */ or *Flavivirus* strains that extensively shares common lesions with *Rift Valley fever* ,*Wesselsbron* ,*Cache valley virus* / or and *Akabane*viruses.

RETRACTED

**Virtual Slides:**

The virtual slide(s) for this article can be found here: http://www.diagnosticpathology.diagnomx.eu/vs/13000_2014_223

## Background

In recent years, with the importation of sheep from abroad, the prevalence of many diseases, especially abortion diseases, has increased in Iran. Surveys on abortion diseases in domestic sheep have been carried out, but most were restricted to *brucellosis, campylobacteriosis, coxiellaburnetii, salmonellosis, leptospirosis*, *neosporosis*, *toxoplasmosis* and other diseases [1-7].

Nevertheless, determining the viral cause of abortion in ovine is obscure, but can be improved with the proper sampling and testing, good communication between veterinarians and diagnostic labs and awareness of the current disease situation in a certain area through authorities’ notification. Therefore, pathologists and field veterinarians who play a very significant role in diagnosis and control should be kept up to date regarding the spread of individual viruses into new geographic areas. On the other hand, despite the importance of fetal viral infections in both humans and animals, many questions regarding mechanisms of transplacental transmission, virus spread within the fetus and the consequences of infection for target cells and the fetus as a whole remain unanswered [8-10]. Whereas, the pathways of virus infection of the fetus and potential protective mechanisms, notably exerted by the innate immune system, are poorly understood despite the fact that transplacental virus infections account for considerable mortality and morbidity in both animals and humans [11].

Pathologic studies can help to confirm the clinical diagnosis and further the understanding of the disease pathogenesis and are very useful in outbreak investigations [12]. Outbreaks of congenital abnormalities in fetal or neonatal ruminants have been related to exposure of pregnant dams to a number of viruses, including *pestiviruses*,*bunyaviruses*, flaviviruses and *arboviruses*, such as *Bluetongue* (BT), *Border disease virus* (BDV) *Wesselsbron* (WSL), *Rift Valley fever* (RVF), *Cache valley virus* (CVV) and *Akabane viruses* (AKV) [13-16]. These abnormalities included stillbirths, mummified fetuses, defects of the central nervous system and musculoskeletal problems. Moreover, the most defects, such as hydranencephaly, hydroencephaly, porencephaly and arthrogryposis and cerebellar hypoplasia, are usually associated with infection with mentioned viruses. In parallel, porencephaly and cerebellar hypoplasia among other congenital anomalies were described in aborted or newborn calves to cows experimentally infected with *Wesselsbron disease* [17]. One report of hydranencephaly and arthrogryposis in sheep infected with *Wesselsbron disease* and *Rift Valley fever viruses* was described by [18], and also, in Akabane disease, necropsy findings of the aborted fetuses are mainly reported in the brain and include microcephaly, hydrocephalus, porencephaly and hydranencephaly [19,20].

RETRACTED

On the other hand, based on experimental and clinical studies performed by researchers, the histological hallmarks of most viral infections in the CNS are neuronal degeneration, perivascular cuffing by inflammatory cells and glial reactivity. Neuronal injury is characterized by central chromatolysis and swelling that progresses to necrosis. The inflammatory reaction is typically non-suppurative and perivascular cuffs mainly consist of lymphocytes, with fewer plasma cells and macrophages, and proliferating vascular adventitial cells. Focal or diffuse microgliosis and formation of glial nodules are characteristic features of viral infections [21,22]. According to these studies*,* viral encephalitis is usually part of a systemic infection rather than the agent having a predilection for neural tissue; however, some viruses are neurotropic and a few multiply within, and cause damage to, the nervous system. Nevertheless, most infections are haematogenous, but some viruses use the fast axoplasmic transport system in nerves to assist invasion [23].

In parallel, RVF virus-induced nonsuppurative encephalitis has been reported in natural infections in human beings and in experimentally infected gerbils and certain strains of rats, but the pathologic characterization of the central nervous system (CNS) lesions has not been described in RVF virus-infected ruminants. In a study, Weiss reported viral encephalitis in two lambs born to ewes vaccinated [24], and in other study, Maar et al. described a case of nonsuppurativeencephalitis in a RVF patient [25]. Another case with encephalitis and retinitis was described by Alrajhi et al. [26], in these patients, the histopathological lesions in brains were characterized by focal necroses associated with an infiltration of round cells, mostly lymphocytes and macrophages, and perivascular cuffing [27]. The aim of the study was to the neuropathological diagnostic features of naturally occurring, a suspected viral infection in the aborted and stillbirth lambs in North of Iran.

RETRACTED

## Methods

### Ethics statement, animals and area

All experiments described in this study were performed in full accordance with the guidelines for animal studies released by the National Institute of Animal Health. The present study was carried out in the different area located in Mazandaran province in the north of Iran (Including the cities of Amol, Ghaemshahr, Neka and Larijan). The number of pregnant sheep in farms varied from 15 to 400. We visited ewes ranches with an abortion rate over 50% for the past 1 year (From February 2012 to March 2013). Whereas, more than 50% of the flocks had experienced abortions, stillbirths and deformities of newborn lambs, but the adult sheep were not affected. Moreover, the sheep flocks comprised mainly indigenous breeds, such as White Mountain Sheep, Brown Mountain Sheep, Zel Breed Sheep and Black headed Mutton.

### History of the outbreak and blood sampling

A total of 650 aborted fetuses including 793 pregnant ewes were studied from 8 flocks at different area in the Mazandaran province during the period of 2012–2013. In some cases, the blood samples from sheep and aborted fetuses were randomly collected from four different locations around Mazandaran province. After coagulation, sera were separated by centrifugation and stored at -20°C until serological testing. But, the results were negative for the detection of *Brucella* spp., *Listeria* spp., *Campylobacter* spp., *Mycoplasma* spp and other infectious agents such as viral, fungal and parasitic.

### Clinical samples and tissue collection

Following macroscopic examination, brain and spinal cord were removed from each fetus. However, the condition of some of the fetuses was such that not all tissues could be collected. Systematic necropsy was performed to collect tissues, and all gross findings were recorded at necropsy by the pathologist. Furthermore, not all tissues were available from each case because the studied abortions occurred under natural conditions, where predation or degree of autolysis resulted in the failure to submit all tissues.

### Histopathological analysis

Tissues collected at necropsy were processed and embedded in paraffin after 48–72 hours of fixation in neutral-buffered 10% formalin. Tissue was sectioned at 5 μm, stained with hematoxylin and eosin, and examined for lesions by light microscopy. Where the brain was available, 14 different sections (from cerebral lobes to medulla oblongata, including cerebellum) together with cervical, thoracic, lumbar and sacral spinal cord segments were studied. Finally, unfortunately, according to the existing facilities at the university, we conducted a limited number of necropsies of aborted fetuses.

RETRACTED

## Results

In the most cases, arthrogryposis was the most common musculoskeletal defects (Figure 1). At postmortem examination significant gross changes were seen in the brains. Malformations of the brain included unilateral or bilateral internal hydrocephalus, characterized by dilated ventricles/or destruction of adjacent neuroparenchyma but still distinguishable gray and white matter; and hydranencephaly (Figure 2), which characterized by segmental or complete loss of the cerebral cortex without discernable gray and white matter; and cerebellar hypoplasia was severe (Figure 2), so that only the brain stem, including pons and medulla oblongata were distinguishable. Porencephalies of the brain stem and gray and white matter of the brain were found in some animals, so that the subcortical cavitations throughout both cerebral hemispheres were also noted (Figure 3). No abnormalities were seen in other tissues.

**Figure 1:** **Lamb born dead with severe arthrogryposis (persistent flexion of the joints): arthrogryposis is one of the congenital abnormalities associated with viral infection.**

**Figure 2:** **Subcortical cavitation (hydranencephaly) in the brain of a lamb infected with viral agent (yellow arrow) together with a severe cerebellar hypoplasia (blue arrow).**

**Figure 3:** **Gross examination of the infected lamb brain with porencephaly in the occipital lobe: a large porencephalic cavitation, which involving a cavity filled with cerebrospinal fluid (CSF).**

In our study, microscopic lesions are mostly confined to throughout the brain and the white and/or gray matter of the brain stem, particularly the pons and the medulla oblongata, and the spinal cord, but, in some cases, CNS lesions mainly identified in the cerebral hemispheres, periventricular areas, midbrain, cerebellum, brainstem and occasionally in the spinal cord. Furthermore, the distribution and severity of lesions in the brain varied among multifarious cases.

Microscopically, inflammation in the CNS characterized by a lymphoplasmacytic*,* mainly perivascular, infiltration of the gray and white matter in most investigated brain areas. Perivascular cuffs ranged from multifarious layers of mononuclear cells. In parallel, encephalitic changes were detected in most aborted fetuses. In these cases, a mild to moderate non-suppurative encephalitis, characterized by foci of perivascular cuffing with mononuclear cells, predominantly lymphocytes, was observed (Figures 4 and 5). The perivascular cuffing was generally associated with a mild to moderate gliosis (focal or diffuse), these changes were most prominent in the cranial brain regions and occasionally the caudal brain regions (pons and medulla). On the other hand, glial nodules (Figure 6) formed predominantly in the mesencephalon, thalamus, hippocampus, pons and medulla oblongata. Nevertheless, mild-to-moderate focal-to-multifocal gliosis associated with acute neuronal necrosis was observed for most cases (Figure 6). Additionally, Virchow–Robin spaces were expanded by cuffs of lymphocytes and plasma cells, admixed with fewer histiocytes and neutrophils. Moreover, multifocal hemorrhages were seen in several cases. These lesions varied in age within each case and between cases.

RETRACTED

**Figure 4:** **Brain; the aborted ovine fetus, naturally infected by viral infection.** Marked lymphoplasmacytic infiltration of Virchow-Robin space (Nonsuppurative encephalitis). H&E .200x and 400x. Bar = 100 and 10 μm.

**Figure 5:** **Brain; the aborted ovine fetus, naturally infected by viral infection.** High-magnification view of perivascular inflammatory infiltrate. Numerous lymphocytes and plasma cells expand the Virchow-Robin space. Endothelial cells are hypertrophied. H&E, 600x. Bar =10 μm.

**Figure 6:** **Photomicrographs of a section of the brain from an ovine fetus; There is severe multifocal gliosis and a focus of gliosis and increased cellularity; H&E .200x and 400x. Bar =100 and 10 μm.**

On the other hand, the most common lesions observed in all infected fetuses which studied were multiple small to large areas of microcavitation/or cyst (Figure 7). These cavities , typically were most common in the cortex. In some cases, in the CNS of aborted fetuses, there was mild to moderate cavitation of the cortex and subcortical white matter (Figure 7). Also, in others, severe cavitation was also observed in the white matter of the cerebellar and cerebellum and also in the adjacent gray matter and cervical spinal cord. However, mild cavitation was also observed in the pons, and lumbar spinal.

**Figure 7:** **Photomicrographs indicate the serial sections of the brain from an ovine fetus.** There are many foci of mild to severe microcavitation. H&E 200x, and 600x. Bar =100, and10 μm.

In some areas, acute neuronal necrosis (Including the eosinophilic/or hypereosinophilic cytoplasm with nuclear pyknosis (ischemic cell changes) and central chromatolysis were mainly in the cortex, subcortical and brainstem regions (Figure 8), and also, in some fetuses, cellular necrosis were observed in the thalamus and temporal cortex in aborted fetuses. In these lesions, degenerating neurons and necrosis can be found, but any nuclear or cytoplasmic inclusions are not observed. The most consistently involved regions are cerebral gray matter and brainstem, closely followed by leptomeninges, as well as, in particular, necrosis neurons were observed in the ventral horns of spinal cord (Figure 9) and mainly were found in arthrogryposis fetuses. In the more severe cases, cerebellum is also involved. Whereas, in most fetuses, there were multiple and discrete foci of cortical necrosis, with loss of the neuropil, increased prominence of blood vessels, gliosis, and microcavitation.

RETRACTED

**Figure 8:** **Micrograph of the superficial cerebral cortex: Slides are from an aborted fetus with nonsuppurative encephalitis.** Note the severe acute neuronal necrosis acute with nuclear pyknosis. Photomicrograph shows a focal gliosis associated with eosinophilicneuronal necrosis. H&E 200x, 400x and 600x. Bar = 100, 10 μm and10 μm, respectively.

**Figure 9:** **Spinal cord; ovine, fetus: Histopathologic analysis disclosed severe neuronal necrosi** ***s o*** **f ventral horn of the spinal cord together with intraspinal hemorrhage.** H&E 200x, and 600x. Bar =100, and10 μm.

The affected blood vessels were lined by hypertrophied endothelial cells and sometimes perivascular edema (Figure 10). The edema was severe in some areas and resulted in marked loosening of the neuropil, resulting in the formation of cavitations. These lesions had variable distribution among the cases and among the various sections of brain regions in each case.

**Figure 10:** **Brain; ovine, fetus: All sections were taken at the different magnification.** There are many foci of perivascular edema surrounding blood vessels together with congested blood vessels and increasedparenchymal cellularity*.* H&E .200x and 400x 600x. Bar =100 and 10 μm.

Briefly ,histopathologic findings in the brain and spinal cord included hyperemia, hemorrhage, non-suppurative encephalitis*,* mononuclear perivascular cuffing, multifocal gliosis, microcavitation,central chromatolysis (Figure 11), neuronal degeneration and necrosis, perineuronal and perivascular edema and necrotic neurons in ventral horn gray matter of spinal cord were present in the all regions of the brain and spinal cord.

**Figure 11:** **A high magnification micrograph of the midbrain with central chromatolysis visualized using hematoxylin and eosin staining (White arrow).** The necrotic cells in the image are those that appear swollen (Yellow arrow). H&E 600x. Bar =10 μm.

## Discussion

Evaluating the areas at risk for the introduction of a new pathogen is challenging. Nevertheless, given the possibility of severe consequences on public and animal health associated with the introduction of a pathogen such as viral infections, the veterinary experts require suitable information on where and how to target surveillance and preventive actions [28,29].

RETRACTED

Based on available data, few studies have been carried out to investigate neuropathological changes after viral infection in the aborted sheep fetuses and also, it is not known why these aborted fetuses demonstrated a different extent of viral infection. Therefore, in parallel, histopathology has been utilized as the gold standard for diagnosis of viral infection, it is well recognized that false-negative results can occur based on the uneven distribution of lesions, particularly in clinical biopsy [30-33].

Previous studies have shown that the most fetal infections with viral causes result in persistent subclinical infection, fetal death, or defects such as cerebellar hypoplasia, hydranencephaly, internal hydrocephalus, microencephaly, and porencephaly. Therefore, these observations are similar to those described in our study. Nevertheless, a number of viruses, including *pestiviruses*, *bunyaviruses*, *flaviviruses* and*arboviruses* are as a teratogenic causes, such as RVF, WSL, CVV, AKV, BTV and pestiviruses like *border disease virus* (BDV) [34-36]. All these virus infections show similar gross findings including cerebellar hypoplasia, por- or hydranencephaly and skeletal malformations like brachygnathia and arthrogryposis of in utero-infected neonates [36-38]. Our results revealed that these malformations occurred in similar high percentages in aborted sheep fetuses with and without CNS inflammation. Cerebellar hypoplasia, porencephaly and hydranencephaly represented the most frequently detected malformations in aborted fetuses together with skeletal malformations like arthrogryposis. In addition to the gross lesions,porencephaly was also detected by light microscopy mainly in the cortex and subcortical white matter. In severe cases, the white matter of the cerebellar and cerebellum was also affected by formation of such cavities. In humans, the occurrence of multiple cysts in the brain due to a hypoxic-ischemic pathogenesis has been described. This entity is termed multicystic encephalopathy [16,39]. The pathological changes associated with viral infection in ruminants seem to fit the description of multicystic encephalopathy.

While a variety of exogenous and endogenous substances are capable of inducing an inflammatory response, a useful principle of neuropathology is that bacterial infections are associated with suppurative inflammation while viral infections are associated with nonsuppurative inflammation [40,41]. Accordingly, the nonsuppurative encephalitis in the aborted ovine fetuses in the present study has the histological hallmarks of a viral infection of the central nervous system: neuronal degeneration and necrosis, reactivity of the glia, and perivascular cuffing with lymphocytes and histiocytes. Furthermore, studies indicated that the variations in the histopathological characteristics of the inflammatory response were detected between animals and anatomical sites and malacia was the most commonly seen feature, but infiltrative or vascular patterns, with malacia, were also detected. Most of these reports however, were based on experimental lesions resulting from the injection of virus into the CNS. Although the pathological investigations of viral encephalitis vary somewhat depending on the specific infectious agent and the immunologic status of the aborted fetuses, most viral infections of the CNS are characterized by a triad of findings including perivascular chronic inflammation, microglial nodules, and neuronal necrosis. Therefor, the mentioned cases are in agreement with our study, moreover, expressed lesions were observed in many samples of our study, and also, the distribution of these findings as well as the presence of characteristic intranuclear or intracytoplasmic viral inclusions can lead to a specific diagnosis in an appropriate clinical setting [42]. Ancillary techniques, including immunohistochemistry (IHC), in-situ hybridization (ISH), or polymerase chain reaction (PCR) amplification, are useful in some settings. These cases are, in contrast, with our observations that not were detected intranuclear or intracytoplasmic viral inclusions in the aborted fetuses.

RETRACTED

In general, in most conducted studies with viral agents on the aborted ovine fetuses, histologic lesions consisted the focal/or multifocal nonsuppurative encephalitis together with the areas of necrosis and loss of the neuronal and motor neurons, cavitation, gliosis ,perivascular and perineural edema at various neuroanatomic sites of the brain and spinal, therefore, in parallel ,based on our study, the mentioned lesions are similar to those described [22,43-47]. Based on these findings, the gross and histologic examination of the brains appears to be important, and viral evaluate may be useful in the postmortem investigation of fetuses with a history of clinical signs referable to the brain.

## Conclusions

In conclusion, therefore, we believe that the histopathological pattern using detected in this study could be associated with either viral infection and or mainly by a *Bunyavirus* / or *Flavivirus* strains that extensively shares common lesions with rift valley fever, WSL and CVV. The true sources of these infections are not known, however, a link between the infected sheep and the condition described here could be suggested. Additional data on these cases are not available because much time has elapsed since it occurred. However, from the history and diagnostic findings on these cases, the etiologic role of *Bunyavirus* / or *Flavivirus* families are a plausible conclusion, thus making these cases the first well-documented evidence of the occurrence of these condition in Iran. And because of the known neurotropism and histologic description of non suppurative encephalitis in viral–infected fetuses, these agents were considered a possible etiologic agent.

RETRACTED

Finally, our study suggested that the aborted/and or infected sheep fetuses are fully susceptible to viral infections and may even develop neurological disease upon natural inoculation of mentioned pathogens. To our knowledge, these are the first direct evidences of the susceptibility to viral causes of aborted fetuses in the north of Iran.
